# Construction of a Public Service Cloud Platform for Disabled People Based on the Big Data Management Model of the Internet of Things

**DOI:** 10.1155/2022/3153454

**Published:** 2022-05-11

**Authors:** Xiaoyan Liu, Guiyang Chang

**Affiliations:** ^1^School of Teacher Education, Weifang University, Weifang 261021, Shandong, China; ^2^General Affairs Department, Weichai Heavy Machinery Co., Ltd, Weifang 261108, Shandong, China

## Abstract

With the continuous development of social economy and the continuous improvement of people's ideological level, the state and social people have given more and more care and assistance to the disadvantaged group of disabled persons. The construction of a public service cloud platform for the disabled is one of the important measures to protect the human rights of the disabled and improve the lives of the disabled. According to the statistics of the China Disabled Persons' Federation, since the twentieth century, with the acceleration of the equalization of basic public services and the establishment of urban and rural social security systems, a practical and effective public service system for the disabled has made leaps and bounds. The construction of the cloud platform for public services for the disabled is an important branch of the construction of the public service system for the disabled. However, due to the late development of the construction of the cloud platform for public services for the disabled in China, it is not perfect, and there are still some problems to be solved. This paper mainly studies the public service cloud platform for the disabled based on the big data management model of the Internet of Things. Based on this research theme, this paper conducts a service response efficiency test for the disabled provided by the disabled public service cloud platform based on the big data management model of the Internet of Things. It concluded that the public service cloud platform for the disabled based on the big data management model of the Internet of Things has improved the response efficiency of providing services for the disabled by 57%.

## 1. Introduction

Persons with disabilities refer to vulnerable people who are deficient in certain functions or organizations of the human body structure compared with those of the able-bodied. The physical defects of the disabled make it impossible for the disabled to participate in the social production and life activities that the able-bodied can carry out. This can easily lead to the disadvantaged social status of the disabled. Therefore, vulnerable groups such as the disabled should be cared for and helped by the whole society. The establishment of a public service system for persons with disabilities is an important measure taken by the state and society to protect the basic human rights of persons with disabilities and provide them with more care and assistance. The public services for the disabled mainly include the following aspects: the first is to protect the basic right to survival of the disabled and meet their basic living needs; the second is to protect the disabled's right to life and health; and the third is to protect the disabled's right to life development, such as promoting their employment and education. Different from other types of public services, public services for the disabled have high fairness and charity. The public service cloud platform for the disabled refers to a more convenient and efficient public service platform built for the disabled relying on modern cloud technology. Since the development of China's public service cloud platform for the disabled is not fully developed, there are still many problems to be solved. Therefore, it is necessary to continuously explore and research more advanced technologies and models that can be applied to the construction of public service cloud platforms for persons with disabilities. IoT big data management mode is a new data management mode based on IoT technology, with strong data and information management functions. This paper mainly studies the construction of a cloud platform for disabled public services based on the big data management model of the Internet of Things.

The innovation of this paper is as follows. (1) The big data management mode of the Internet of Things is introduced, and the construction of the public service cloud platform for the disabled is explored based on the big data management mode of the Internet of Things. (2) It has built a public service cloud platform for the disabled based on the big data management model of the Internet of Things. It also tested the response efficiency of the platform in providing services to persons with disabilities and came to valid conclusions.

## 2. Related Work

In recent years, there have been many research studies related to the big data management model of the Internet of Things in academia. Among them, Din S studied the application of IoT big data management model in the field of healthcare. He proposed a new architecture for IoT big data management specifically for aggregating and processing real-time data in the healthcare domain [1]. Rajput S studied the application of IoT big data management model in Industry 4.0. He proposed that the IoT big data management model plays an important role in data and information management in Industry 4.0. It is one of the most reliant data management enablers in industry [2]. Sarosh P's research focused on the application of IoT big data management models in the field of medical big data analysis. He proposed an IoT big data management framework for medical big data [3]. Dong J's research is about the application of IoT big data management model in urban road network road maintenance. He developed a pavement management system and road maintenance management architecture based on the big data management model of the Internet of Things [4]. Manogaran G's research proposed a new IoT big data management architecture for storing and processing scalable sensor data for healthcare applications [5]. Sood S K's research proposed an intelligent flood monitoring and early warning architecture based on the big data management model of the Internet of Things. This architecture classifies geographic areas into hexagonal networks for efficient installation of energy-efficient IoT devices [6]. However, the studies have a common disadvantage; that is, the research process is complicated and difficult to operate. It takes a lot of time and effort to invest.

## 3. Construction Method of Public Service Cloud Platform for Disabled Persons

### 3.1. IoT Infrastructure

IoT is a powerful intelligent network architecture. Its basic concept is to connect various things ubiquitous in the human living environment through unique solutions, and it processes and analyzes relevant data and information [7]. The Internet of Things can automatically collect and analyze data information on the environment and things in a full range and anytime and anywhere through a variety of sensing devices and build a data management service platform based on this. This makes people's social life and production decisions more intelligent and informatized through different application systems [8]. The infrastructure of IoT is shown in Figure 1.

Among them, the perception layer is mainly used to collect physical information. The perception layer mainly includes two types of facilities: the perception terminal and the field network. The sensing terminal has sensing, computing, and communication capabilities. The network layer is the information backbone of the Internet of Things. It includes various IP factory area networks provided by communication operators, including both wired and wireless networks. And because wireless networks can be configured and managed more flexibly, high-speed wireless networks are more suitable communication media for IoT applications [9, 10]. The management layer includes the platform layer, which integrates the management, control, and operation of terminals and assets. It includes integration frameworks, IoT middleware, and cloud computing platforms. The application layer is the interface between the IoT and the user. It is combined with industry needs to realize the intelligent application of the Internet of Things. The powerful functions of the Internet of Things make it widely used in many fields, such as media operations, environmental monitoring, infrastructure management, energy management, healthcare systems, and buildings and smart homes [11, 12].

### 3.2. IoT Big Data Management

The Internet of Things is a huge intelligent network architecture formed by combining massive sensing devices with the Internet. In the Internet of Things, massive sensing devices continuously collect data and send it to the data center. With the continuous development of perception technology and network technology, the collected data present massive characteristics, forming the Internet of Things big data [13]. The extension of the Internet of Things is very extensive, and the data in various application fields have different characteristics. It can be summed up as shown in Table 1.

It can be seen from Table 1 that IoT big data in different fields has significantly different characteristics. However, IoT big data has the common characteristics of multisource heterogeneity, mass, spatio-temporal correlation, and real-time. Moreover, IoT data also has a certain life cycle. The life cycle of IoT refers to a complete process of processing and analyzing IoT big data [14], as shown in Figure 2.

Among them, the query request in the Internet of Things mainly refers to the request for local real-time data based on monitoring purposes and the retrieval of global data based on specific services. Data generation refers to the generation of perception and transmission data, which are regularly pushed and reported for applications within the IoT framework that are interested in these data [15, 16]. Data collection is when sensors and smart devices within the IoT may store or report data to their management components at certain intervals. The collected data may be further sifted and processed in the network and fused into a more efficient and compact form for dissemination. Data fusion technology is used to aggregate, combine, and compress the amount of data for storage and transmission in real time. Data delivery means that the process results generated after data are filtered and aggregated by a certain unit in the Internet of Things may need to be further sent to other modules. It is either used as the final response for storage and in-depth analysis. Data preprocessing refers to removing redundant data in advance and integrating data from different data sources into a unified schema for storage in the process of data processing. The data storage and archiving phase is the efficient storage and update of data, which can ensure high availability of data. Data analysis involves the retrieval and analysis of stored and archived data. It uses historical insights to predict future trends or detect abnormal data to trigger other actions. As shown in Figure 2, there are three possible ways that data flows in IoT. One is for queries within local subsystems. Data are generated, processed, and delivered within the network. The second is for global or real-time queries. Data start in production, then are collected, and then they are sent to integration and delivery The last one is further aggregation of data. It includes data preprocessing, persistent storage, and archiving, followed by in-depth processing and analysis [17].

There are three different levels of management and analysis of data in IoT. They are a single data source, a single data point with multiple data sources, and multiple data points from multiple sources. IoT big data management frameworks must support data at different levels. In addition, it needs to support real-time and offline processing modes of data. In addition, the framework must be flexible to support new data sources so that they can be seamlessly integrated into existing systems. IoT big data management frameworks also allow various different entities to analyze and manage the data that needs to be processed with varying degrees of flexibility. According to the life cycle of IoT data proposed [18], the IoT big data management framework mapped to each stage of the data life cycle is shown in Figure 3.

### 3.3. IoT Big Data Management Real-Time Processing Model RVIM

In this paper, two main approaches to deal with the big data VIoT of the Internet of Things are considered. One is real-time (online) mode, and the other is batch (offline) mode. Next, this paper discusses these two modes separately and gives the mathematical models of the two modes. In real-time mode, the IISP will immediately process the VIoT request when it receives it [19]. If multiple VIoTs arrive at the same time, they will be processed one by one in the queue. Earlier we defined the gross profit for the IISP to accept a VIoT request. Here, we give the cost required by IISP to map a VIoT request:

(1) $$\begin{array}{c} C\left(I^{U}\right)=\overset{x}{\underset{s}{\sum }}P\overset{\theta }{\underset{t}{\sum }}R_{t}\left(S^{v}\right)+\overset{y}{\underset{g}{\sum }}t. \end{array}$$

In the equation, the variables and *R*_*t*_ represent the unit cost of resources of class *t* on PSN and PG, respectively. IISP receives a single VIOT mapping as follows:

(2) $$\begin{array}{c} P\left(I^{V}\right)=R\left(I^{v}\right)-T\left(I^{v}\right). \end{array}$$

The goal of this article is to maximize the profits of the IISP. Therefore, the real-time VIoT mapping model (RVIM) proposed in this paper is as follows:

(3) $$\begin{array}{c} f=\max P\left(I^{v}\right). \end{array}$$

Among them, the capacity constraint is as follows:

(4) $$\begin{array}{c} \overset{s}{\underset{v}{\sum }}x_{p}^{s}R_{t}\left(s^{v}\right)\leq A_{t}\left(S^{P}\right),\\ \overset{g}{\underset{v}{\sum }}y_{t}^{v}\left(g^{v}\right)\leq A_{t}\left(g^{P}\right). \end{array}$$

Finally,

(5) $$\begin{array}{c} \sum y_{g}^{v}\leq A_{t}\left(S^{p}\right). \end{array}$$

The capacity constraints are to ensure that the various resources on each PSN and PG are adequately allocated to the request. Among them, *A*_*t*_(*s*^*p*^) and *A*_*t*_(*g*^*p*^) represent various resources currently available on PSN and PG, respectively.

The virtual path constraints are as follows:

(6) $$\begin{array}{c} \underset{p\in L_{o}}{\sum }fe_{p}^{v}=QR_{b}\left(e^{v}\right). \end{array}$$

The domain constraints are as follows:

(7) $$\begin{array}{c} \overset{s}{\underset{p}{\sum }}x_{v}^{s}=1,\;\forall s^{v\in }s^{v}, \end{array}$$

which is

(8) $$\begin{array}{c} \underset{g^{p}}{\sum }y_{p}^{v}=1,\forall_{g}^{v}\in G^{v}. \end{array}$$

There is also an important constraint in the IoT big data management model, that is, the geographical location constraint.

First,

(9) $$\begin{array}{c} x_{s}^{v}=s^{p}\cap \beta \left(s^{v}\right). \end{array}$$

Next,

(10) $$\begin{array}{c} x_{p}^{v}=g^{p}\cap \vartheta \left(g^{v}\right). \end{array}$$

Combined with the content, there are a total of 6 constraints in the specific expansion. The virtual path constraint ensures that all virtual sensing nodes VSN in *I*^*v*^ must be mapped to physical sensing nodes [20]. Also, the domain constraint ensures that all virtual gateways VG in *I*^*v*^ are mapped to physical gateways PG. In the RVIM model, VIOT is accepted only if all elements of the VIoT can be mapped; otherwise, it is rejected. Although the goal of the RVIM model is to map individual VIoTs, it is still possible to build a waiting queue to store all VIoTs. It can also be sorted according to the size of the VIoT, the additional cost provided by the VIoT, fairness, priority, and other factors. A rejected VIoT can be inserted into a queue waiting to be rescheduled [21]. In this RVIM model, solving the above model is solving the mapping problem of VSN, VG, and VLs at the same time. This single-stage mapping strategy avoids the hassle of coordination required for multistage mapping problems.

While the RVIM model is capable of processing submitted requests in real-time, the RVIM model lacks forward-looking. It may not be the best mapping strategy in the long run. For example, when the RVIM model performs the mapping immediately upon the arrival of the first VIoT request, in order to minimize the cost or maximize the profit of the mapping, the two perception nodes in the VIoT will be simultaneously mapped to the PSN on the left or right. Regardless of which PSN the first VIoT is mapped to, when the second VIoT arrives, the IISP will reject it due to insufficient remaining resources. However, when these two VIoT requests are processed simultaneously, they can be successfully mapped. In conclusion, mapping all elements of the first VIoT to the same physical node is probably the best option for the current situation. However, this strategy is not optimal in the long run. Therefore, in order to solve this “myopia” problem, it proposes a batch VIoT mapping (BVIM) model. In this model, several VIoT requests are grouped together and processed simultaneously, rather than one after the other as in the RVIM model. This strategy avoids the imbalance of resource utilization and further improves the profit of IISP [22].

The BVIM model is as follows:

(11) $$\begin{array}{c} \pi_{w}=\max f\pi \overset{k}{\underset{j=1}{\sum }}\pi_{j}P\left(I_{j}^{v}\right). \end{array}$$

The capacity constraints of the BVIM model are as follows:

(12) $$\begin{array}{c} \overset{k}{\underset{j=1}{\sum }}\pi_{j}\leq A_{t}\left(S^{P}\right), \end{array}$$

which is

(13) $$\begin{array}{c} \overset{k}{\underset{j=1}{\sum }}\pi_{j}\leq A_{b}\left(e^{P}\right). \end{array}$$

The virtual path constraint is then

(14) $$\begin{array}{c} \pi_{j}\underset{e}{\sum }f_{p}^{v}=\pi_{j}Q_{p}^{v}R_{b}\left(e^{v}\right). \end{array}$$

The domain constraints are

(15) $$\begin{array}{c} \underset{s}{\sum }x_{v}^{s}=\pi_{j},\forall s_{j}^{v}\in s_{v}^{j}. \end{array}$$

Finally, the geolocation constraints are

(16) $$\begin{array}{c} x_{s}^{v}=s^{p}\cap \mu \left(s^{v}\right). \end{array}$$

## 4. Service Response Efficiency Test Experiment of the Disabled Public Service Cloud Platform

### 4.1. Experimental Design and Platform Construction

This chapter studies the service response efficiency of the disabled public service cloud platform in the IoT big data management model. First, based on the big data management model of the Internet of Things, this paper builds a public service cloud platform for the disabled and then tests the service efficiency of this cloud platform. According to the test results, it evaluates the efficiency and effect of the disabled public service cloud platform based on the IoT big data management model to provide services for the disabled.

First of all, it is necessary to build a public service cloud platform for the disabled suitable for the research of this paper according to the big data management of the Internet of Things. The public service cloud platform for the disabled built based on the big data management model of the Internet of Things in this paper is shown in Figure 4.

It can be seen from Figure 4 that the architecture of the public service cloud platform for disabled persons based on the big data management model of the Internet of Things is relatively complete, and the framework structure is also closely related.

### 4.2. Service Efficiency Test of the Public Service Cloud Platform for the Disabled

After building a public service cloud platform for the disabled based on the big data management model of the Internet of Things, the platform can be run and the service efficiency provided by the public service cloud platform for the disabled can be tested. The test was conducted in the following way: first, 4 persons with disabilities were randomly selected to participate in this test. They will use the platform to obtain the services they need and record the response time of the disabled public service cloud platform based on the big data of the Internet of Things to provide the four disabled people with the services they need. And it was compared with the response time of similar services provided by other public service cloud platforms for the disabled, so as to compare and calculate the efficiency of the public service cloud platform for the disabled based on the big data management model of the Internet of Things to provide services for the disabled.

First, the services provided by the public service platforms required by the four disabled persons are shown in Table 2.

Four test results of the response time and corresponding efficiency required to provide these services on the common disabled public service cloud platform are shown in Figures 5 and 6.

From Figures 5 and 6, it can be concluded that the average response times of the common disabled public service cloud platforms for these four services are 3.5 minutes, 4.5 minutes, 4.5 minutes, and 2.5 minutes, respectively.

The four test results of the response time of these four services provided on the public service cloud platform for the disabled based on the IoT big data management model are shown in Figures 7 and 8.

It can be seen from Figures 7 and 8 that the average response time of the four services provided by the cloud platform of public services for the disabled based on the IoT big data management model is 4.5 minutes, 2 minutes, 1 minute, and 1.5 minutes. The average response time is significantly lower than that of common platforms.

To sum up, the conclusion of this experiment can be drawn through calculation: the public service cloud platform for the disabled based on the big data management model of the Internet of Things has improved the response efficiency of providing services for the disabled by 57%.

## 5. Discussion

Due to their physical defects, it is extremely difficult for the disabled to survive and develop in society. In order to maintain social harmony, they also deserve more care and help from the society. The country and society are also constantly exploring how to provide more and better services for the disabled to meet their survival and development needs. The disabled public service cloud platform is a service platform constructed to provide more efficient and convenient services for disabled groups [23, 24].

With the development of social economy, the construction of public service cloud platform for the disabled is also developing continuously. More and more advanced science and technology can play some roles in the construction of the public service cloud platform for the disabled, such as the big data management model of the Internet of Things. This paper mainly studies the construction of a cloud platform for disabled public services based on the big data management model of the Internet of Things.

This paper builds a public service cloud platform for disabled people based on the big data management model of the Internet of Things and tests the response time of this platform for providing services for disabled people. The test results show that the response time of the disabled public service cloud platform based on the big data management model of the Internet of Things has been significantly improved, which means that the response efficiency of the platform for the disabled has also been improved. According to calculations, the response efficiency of the disabled public service cloud platform based on the IoT big data management model for providing services to disabled people is increased by 57%. It shows that the big data management model of the Internet of Things has a positive effect on the construction of the public service cloud platform for the disabled.

## 6. Conclusion

Caring and helping the disabled are conducive to ensuring and promoting social harmony, and building a public service cloud platform for the disabled is one of the important measures to provide care and assistance for the disabled. Based on the big data management model of the Internet of Things, this paper conducts a service response efficiency test of the public service cloud platform for the disabled. The conclusion shows that the public service cloud platform for the disabled built based on the big data management model of the Internet of Things has significantly improved the response efficiency of providing services for the disabled. The research conclusions drawn in this paper have a certain role in promoting the construction and development of the public service cloud platform for the disabled. However, due to the limited research level and conditions, the research of this paper also has some limitations, such as the research method is not innovative enough, and it is relatively simple. It is hoped to do better in the future and contribute more to the construction of the cloud platform for public services for the disabled.

## Figures and Tables

**Figure 1:** IoT infrastructure.

**Figure 2:** IoT big data lifecycle.

**Figure 3:** IoT big data management framework.

**Figure 4:** Cloud platform for disabled public services based on the IoT big data management model.

**Figure 5:** 1st and 2nd service response time and efficiency test results for common platforms. (a) 1st test. (b) 2nd test.

**Figure 6:** 3rd and 4th service response time and efficiency test results for common platforms. (a) 3rd test. (b) 4th test.

**Figure 7:** 1st and 2nd service response time results for the build platform. (a) 1st test result. (b) 2nd test result.

**Figure 8:** 3rd and 4th service response time results for the build platform. (a) 3rd test result. (b) 4th test result.

**Table 1:** Types of IoT data.

Type of data	Type description	Type example
Geographic data	Object geographic attribute description	Size, height, width

Media data	Object media property description	Sound, image, video

Status data	Object physical state description	Temperature, humidity, current

Time data	Object time state description	Occurrence, effective time

**Table 2:** Public services needed by people with disabilities.

	Service type	Difficulty of service
Disabled 1	Seek employment	Difficult
Disabled 2	Receive education	Medium
Disabled 3	Medical insurance	Generally
Disabled 4	Entertainment and relaxation	Easy

## Data Availability

No data were used to support this study.
